The article "A Novel Approach for Feature Selection and Classification of Diabetes Mellitus: Machine Learning Methods" was published in 2022. Journal: Comput Intell Neurosci.

# A Novel Approach for Feature Selection and Classification of Diabetes Mellitus: Machine Learning Methods

**DOI:** 10.1155/2022/3820360

**Published:** 2022-04-15

**Authors:** Roshi Saxena, Sanjay Kumar Sharma, Manali Gupta, G. C. Sampada

**Affiliations:** ^1^CSE Department, Gautam Buddha University, Greater Noida, India; ^2^Cedargate Technologies, Kathmandu, Nepal

## Abstract

An active research area where the experts from the medical field are trying to envisage the problem with more accuracy is diabetes prediction. Surveys conducted by WHO have shown a remarkable increase in the diabetic patients. Diabetes generally remains in dormant mode and it boosts the other diseases if patients are diagnosed with some other disease such as damage to the kidney vessels, problems in retina of the eye, and cardiac problem; if unidentified, it can create metabolic disorders and too many complications in the body. The main objective of our study is to draw a comparative study of different classifiers and feature selection methods to predict the diabetes with greater accuracy. In this paper, we have studied multilayer perceptron, decision trees, K-nearest neighbour, and random forest classifiers and few feature selection techniques were applied on the classifiers to detect the diabetes at an early stage. Raw data is subjected to preprocessing techniques, thus removing outliers and imputing missing values by mean and then in the end hyperparameters optimization. Experiments were conducted on PIMA Indians diabetes dataset using Weka 3.9 and the accuracy achieved for multilayer perceptron is 77.60%, for decision trees is 76.07%, for K-nearest neighbour is 78.58%, and for random forest is **79.8%**, which is by far the best accuracy for random forest classifier.

## 1. Introduction

Diabetes, also known as silent killer, is caused when the level of glucose in the body increases beyond a certain point in the blood. When the glucose in the body remains undigested or is not metabolized properly, levels of sugar in the blood increase. The main source of energy in our body is glucose which is fulfilled through the food we eat generally. A hormone known as insulin absorbs the glucose from the pancreatic cells and creates the energy required for the body. But when the insulin is not produced in sufficient quantity, glucose keeps on accumulating in the blood and hence the level increases. There is no cure for diabetes, but the person can lead a healthy life after following a balanced routine. However, if the proper treatment is not received at an appropriate time, organs of the body like kidneys, nervous system, and eyes, lower limb amputation, and heart problems can deteriorate. Therefore, it is better to predict diabetes as early as possible so that the parts of the body can function properly. Statistics released by WHO have stated that approximately 470 million people in the world were suffering from diabetes till 2019 and approximately 700 million people are likely to suffer from it by 2045. There are three types of diabetes and a prediabetic condition.

*Type 1 Diabetes*. It is when the insufficient amount of insulin is being produced by pancreatic cells and it is injected through outer sources to maintain the body glucose levels. Generally younger people suffer from this type of diabetes.

*Type 2 Diabetes*. It is when the metabolic action of the body is unable to digest the food completely, thus increasing sugar in the blood. Hereditary can also be one of the reasons of this type of diabetes. Older people in the age range of 45–60 years generally suffer from this type of diabetes.

*Gestational Diabetes*. Changes in hormones and high amount of insulin production during pregnancy trigger this kind of diabetes.

*Prediabetes*. This condition is also known as borderline diabetes in which there are high levels of sugar but not up to the level which can be diagnosed as diabetes.

In our paper, we have made use of few machine learning algorithms, that is, decision trees, multilayer perceptron, and random forest, to make predictions for diabetes. Machine learning is a concept which learns from examples and historic data and, based on the study of historical data, predictions are made for futuristic data. Programmers do not need to do programming here as logic is built on the trained data and tested on test data. It is a branch of artificial intelligence where the predictions are made on the basis of experience. It is of the two following types.

*Supervised Learning*. Learning is guided through a trained model. A new model is trained using the given input trained dataset or model and, after the training of the new model, predictions are made.

*Unsupervised Learning*. Learning [1] is done through observation. The algorithm tries to find some specific structure and patterns in the dataset and classifies the data according to the patterns and structural relationships in the dataset.

In this paper, we focus on the comparative analysis of three feature selection methods, namely, correlation attribute selection, information gain, and principal component analysis, for classification of diabetic patients (268) and nondiabetic patients (500) and further comparing K-nearest neighbour, random forest, decision trees, and multilayer perceptron. The performance parameters are precision, recall, accuracy, true positive rate, true negative rate, and area under the curve. The following are the novelties and contributions of our machine learning system:

1. Comparative analysis between the three feature selection methods, that is, correlation attribute evaluation, information gain, and principal component analysis, for predicting diabetic patients and nondiabetic patients
2. Optimizing dataset by rejecting outliers and imputing missing values in the PIMA Indians diabetes dataset
3. Hyperparameter optimization for K-nearest neighbour, random forest, decision trees, and multilayer perceptron and demonstration of improvement in accuracy by 8.4%, 3.9%, 2.27%, and 2.5%, respectively
4. Computation of performance parameters, that is, precision, recall, accuracy, true positive rate, true negative rate, and area under the curve
5. Benchmarking our machine learning system with available methods present in the literature

The remainder of the paper is organized as follows: The Related Work section presents the study of available methods to classify the patients into diabetic and nondiabetic. The Materials and Methods section represents description of feature selection methods, machine learning system, preprocessing techniques, dataset description, tool description, and classifiers evaluation. The Results section discusses the results of all classifiers [2] applied before feature selection, data preprocessing, and tuning of hyperparameters and after the proposed method. The Conclusion section discusses the summary of current work and future work.

## 2. Related Work

In recent years, a good amount of research work has been done to forecast the diabetes using machine learning technique.

Sneha et al. [3] made use of optimal feature selection method to enhance the accuracy of classification methods and showed that Naïve Bayes method is giving the best accuracy, while random forest is giving highest specificity. Hasan et al. [4] made use of correlation, principal component analysis feature selection methods, and ensemble classifiers and achieved the maximum AUC by using ensemble of AdaBoost and Gradient. Data is preprocessed using outlier rejection and calculating the mean and median of misplaced values, data and information standardization, selection of relevant features, and applying 10-fold cross-validation. After running the different classifiers such as K-nearest neighbor, random forest [5], decision trees, and Naïve Bayes, the ensemble of AdaBoost and Gradient boost was found to perform better than all the other classifiers. Tuning of hyperparameters was done using grid search technique. Maniruzzaman et al. [6] applied logistic regression to extract the important features from NHANES diabetes dataset and achieved the result by using random forest classifier. The authors compared accuracy, sensitivity, true positive rate, false positive rate, f-measure, and area under the curve. Kamadi et al. [7] identified the false split points and made use of Gaussian fuzzy membership function to eliminate the false split points. The framework has been tested on PIMA Indian diabetes dataset. Maniruzzaman et al. [8] applied feature reduction technique to reduce the dimensions of dataset. Comparison was made amongst quadratic discriminant analysis [9] and linear discriminant analysis [10] to select the significant features. The authors classified the data using Naïve Bayes [11], logistic regression [12], AdaBoost [13], neural network [7], support vector machines [14], random forest [15], Gaussian process [16], and decision trees [17]. Sisodia et al. [18] made use of various classifiers on PIMA Indian diabetes dataset and showed that Naïve Bayes outperforms every other classifier in terms of accuracy. Genetic programming was used by Bamnote et al. in [19] to first train the model and then test the database for diabetes prediction. Optimal accuracy was achieved using genetic programming as compared to other implemented techniques. It was useful for predicting diabetes at low cost and by taking less time for classifier generation. Perveen et al. [20] discussed ensemble of AdaBoost and Bagging by making use of J48 decision tree for classifying the diabetes. After performing extensive experiments, AdaBoost machine learning outperformed Bagging as well as J48 technique. Robustness was increased by boosting techniques in the prediction of diabetes and Nai-arun et al. [21] classified the data using K-nearest neighbour, Naïve Bayes, decision trees, and logistic regression. In [22], Gaussian process-based classification technique is used by making use of linear, polynomial, and radial-basis kernel and a comparison was drawn against linear discriminant analysis, quadratic discriminant analysis, and Naïve Bayes. Extensive experiments were carried out to find the best working cross-validation protocol. Their experiments revealed that Gaussian process-based classifier [23] along with 10-fold cross-validation protocol is the best classifier for predicting diabetes. In the work of Orabi et al. [24], a system for predicting the diabetes at a particular age was designed by the authors and the system was based on application of decision tree algorithm. The system worked well and gave higher accuracy with decision tree [25] in predicting diabetes at a particular age. Rashid et al. [26] designed a prediction model for diabetes prediction by clubbing two submodules. Artificial neural network was used in the first submodule and fasting blood sugar was used in the second submodule, where the two submodules are clubbed together for predicting diabetes. Decision tree [27] was used to distinguish the signs of diabetes. Mohapatra et al. [28] made use of neural network and carried out testing on divided dataset. The dataset has been divided into training dataset and testing dataset and it was proved that testing data gives the classification accuracy of 77.5% when being divided. Two classifiers of machine learning algorithms, that is, Bayesian regulation and artificial neural network, were used by Alade et al. [29] for training the dataset and avoiding any overfitting in the dataset. Output was displayed via regression graphs. Comparison of both classifiers, that is, artificial neural network and Naïve Bayes, was done by Ali'c et al. [30] and the authors showed that neural network is better than the Bayesian classifier. Depression was identified in type 2 diabetic patients by Khalil et al. [31] by applying support vector machines, probabilistic neural network, fuzzy c-means algorithm, and K-means algorithm. Diabetic retinopathy was detected by Carrera et al. [32] on the basis of digital retinal images. Naïve Bayes, logistic regression, and tenfold cross-validation technique were implemented by Lee et al. [33] to select the best prediction model for identification of type 2 diabetic patients.

## 3. Materials and Methods

### 3.1. Feature Selection

One of the important steps of the proposed method is selection of features. Feature selection [34] is reducing the dimensionality of dataset by selecting the appropriate features from the original feature set based upon some evaluation criteria and eliminating redundancy from the dataset by removing redundant features from the feature set. Suppose that we have a set of features *N* having *n* number of features {*n*_1_, *n*_2_, *n*_3_,…, *n*_*k*_}. Feature selection is the process of selecting *k* relevant features from this feature set. The entire process of selection of features involves subset generation, evaluation, and respective measures to stop and search for procedures for validation.

#### 3.1.1. Correlation Based Feature Selection

Feature selection is selection of significant features for classification purpose. For example, if we have to purchase a house in a particular location, there are *n* numbers of features associated with the house and feature selection method enables us to identify relevant features from the list of features provided, which can help us in having better evaluation. Attributes [35] are evaluated with respect to what is known as target class and Pearson's correlation method is made use of to calculate the amount of correlation between each feature and features of target class. Nominal attributes are considered on value basis and every value pretends to be an indicator.

Features selection extracts a subset of relevant features from the provided dataset depending upon the criteria being evaluated. A set of features are divided into *n* subsets. Sorting of the features is done in ascending order of relevance. Redundancy could be present between a feature vector and its neighbour feature vector. To remove the redundancy between two feature vectors, symmetric uncertainty is used. If two redundant features are present in the dataset, we can remove one of the redundant features, since both of them will give us almost the same result. There are many attributes in the patients records which can be used for diagnosing the medical condition of the patient. Classifier's performance highly depends upon the attribute selection. Good attributes which are relevant to the classification purpose are selected but there should not be any redundancy. Correlation between two attributes is selected through either classical method of linear correlation or another method which is based on information theory. In the classical method of linear correlation, for each pair of (*x*, *y*) coordinates, we have the following coefficient:

(1) $$\begin{array}{c} r=\frac{\sum_{i=o}^{n}\left(x_{i}-{\bar{x}}_{i}\right)\left(y_{i}-{\bar{y}}_{i}\right)}{\sum_{i=o}^{n}\left(x_{i}-{\bar{x}}_{i}\right)\wedge^{2}\sqrt{\sum_{i=o}^{n}\left(y_{i}-{\bar{y}}_{i}\right)}\wedge 2}, \end{array}$$

where *r* is coefficient of linear correlation, *X*_*i*_ is mean of *x*, and *Y*_*i*_ is mean of *y*.

The coefficient lies within the range of −1 and +1. If the value of the coefficient is 0, then variables *x* and *y* are considered to be independent variables. On the other hand, we can make use of entropy as well alternatively. Entropy of variable *x* is defined as follows:

(2) $$\begin{array}{c} H\left(x\right)=\;-\sum_{i=0}^{n}P\left(x_{i}\right){\text{log}}_{2}\left(P\left(x_{i}\right)\right). \end{array}$$

The conditional entropy of *x* given another variable *y* is calculated using the following equation:

(3) $$\begin{array}{c} H\left(\frac{x}{y}\right)=\;-\sum_{j=0}^{n}P\left(x_{j}\right)\sum_{i=0}^{n}P\left(\frac{x_{i}}{y_{j}}\right){\text{log}}_{2}\left(P\left(\frac{x_{i}}{y_{j}}\right)\right), \end{array}$$

where *P* (*x*_*i*_) is probability of all values of *x* and *P* (*x*_*i*_/*y*_*i*_) is posterior probability of *x* given value of *y*.

We can make use of symmetric uncertainty given in equation (4) also to measure the correlation between the attributes:

(4) $$\begin{array}{c} \text{SU}\left(x,y\right)=2\left[\frac{\text{IG}\left(x/y\right)}{H\left(x\right)+H\left(y\right)}\right]. \end{array}$$

If the symmetric uncertainty is 1, that means *x* and *y* are completely correlated.

#### 3.1.2. Principal Component Analysis

It is also one of the feature selection methods which is used to reduce the dimensionality of the feature set. Principal component analysis is a type of feature selection method which is an orthogonal linear transformation where the data is transformed to a new coordinate system in which first coordinate has principal component [36], that is, the greatest variance, second coordinate has second greatest variance, and so on. Our dataset consists of *m* columns and *n* rows; it can be taken as a matrix *X* of *m* × *n* dimensions where each column has a zero empirical mean. Empirical mean is the average mean of every column which has been shifted to zero and the column represents a specific feature from the feature set and rows are the experiment repetitions.

Orthogonal linear transformation [37] is mathematically represented as a set of finite sizes *m* of *n*-dimensional vectors where the coefficients is

(5) $$\begin{array}{c} C_{\left(k\right)}={\left(C_{1},\ldots ,C_{n}\right)}_{k}, \end{array}$$

where each row vector is mapped to scores of principal component's new vector and is represented by the following equation:

(6) $$\begin{array}{c} t_{\left(k\left(i\right)\right)}=x_{\left(i\right)}C_{\left(k\right)}\text{ for }i=1,2,\ldots ,n\text{ and }k=1,2,\ldots ,m. \end{array}$$

Calculating principal component is as follows:

- Ignore the labelled component and take the rest of the dataset as *d*-dimensional
- Mean of every dimension or column of the dataset is calculated
- Covariance matrix of the whole dataset is computed
- Eigenvectors and eigenvalues are computed
- Eigenvectors are sorted in order of descending eigenvalues and *k* eigenvectors with the highest eigenvalues being chosen to form a *d* × *k*-dimensional matrix
- The above computed matrix is used for sample transformation into the new subspace

#### 3.1.3. Information Gain Attribute Selection

Information gain feature selection measures the amount of information about the class which a feature can provide us. Features that are not related to each other do not provide us any information. Features are ranked in descending order on the basis of high information gain entropy. The amount of information provided by a feature is calculated using entropy. Information gain measures reduction in entropy.

Entropy is calculated as follows:

(7) $$\begin{array}{c} E\left(S\right)=\sum_{i=1}^{c}-P_{i\;\log_{2}P_{i}}, \end{array}$$

where *p* is proportion of instances belonging to class.

The higher the entropy is, the lower the level of purity is. The information gain is based on the decrease in entropy after a dataset is split on an attribute.

Information gain is calculated by the following steps:

- Calculate entropy of branch.
- Split the dataset into different attributes and then calculate entropy for each branch. Total entropy of the split is calculated by adding entropy of the branch proportionally.
- Subtract the resultant from entropy as it was before split.
- Net result is the information gain

### 3.2. Machine Learning Algorithms

#### 3.2.1. Multilayer Perceptron

Neural network consists of input layer, output layer, and hidden layers. The input layer accepts the data and we get result from output layer. Hidden layer is present between input layer and output layer. Neural network takes its origin from neural network of human brain. Probabilistic behaviors of neurons in network are similar to neurons in human being. Processing time is quite high in neural networks. It is also known as multilayer perceptron in Weka.

#### 3.2.2. Decision Tree

Decision tree splits the dataset based on certain condition. The first node of the decision tree is called root node and the internal nodes are known as decision nodes where the data gets split and outcome is achieved. Decision trees can be used for regression purpose as well as for classification purpose. It follows a set of if-then and else rules. Different features with instances are classified by root node and the leaves represent the classified result. Every node is chosen by evaluation of information gain amongst all attributes.

Working of decision tree is as follows:

- A tree is constructed by taking its input features as nodes
- Features are selected and the output is predicted from the input nodes with the highest information gain
- The above steps are repeated to form a number of subtrees on those features which were not used in the root node

#### 3.2.3. Random Forest

Random forest is a collection of large number of decision trees. Prediction is made by each and every tree on data samples and best solution is selected by means of voting. The result of every decision tree is averaged which also helps in reducing overfitting. Random forest classifiers can be used for regression as well as classification purpose.

Working of random forest is as follows:

- Random samples are selected from the given dataset
- Decision tree is constructed for every sample and predictions are made from every decision tree
- Every predicted result undergoes voting
- The result which has the highest votes will be the final predicted result

#### 3.2.4. K-Nearest Neighbour

K-nearest neighbour algorithm [38] is a supervised algorithm which can be used for both regression and classification purposes but is mostly used for classification purpose. KNN is also known as lazy algorithm, since it works on stored dataset and, at the time of classification, it makes the prediction on the dataset. It makes the resemblance between dataset stored and new test data which is being fed to it. It classifies the test data based on a similarity with trained data. It is also known as nonparametric classifier, since it does not make any guesses on the underlying data. When the new data is fed to classifier, it makes the resemblance between new data and the data which is quite similar to new data and the new data is assigned to similar categorical data.

How KNN algorithm works: It makes use of similar feature concept to make new predictions. Testing data will be given a value which matches the similar kind of value in trained dataset.

- training and testing datasets are loaded.
- value of the K*-*nearest neighbour is chosen. *K*'s value can be integer.
- For each value in testing dataset, the distance between each row of the trained dataset and test data is calculated. The distance can be calculated using either Euclidean or Manhattan or hamming distance. The distance value is then sorted in ascending order. After being sorted, top k-rows are chosen from the array of distance values. Test points are classified on the basis of most frequent class of the k-rows.

### 3.3. Data Preprocessing Technique

After selecting significant features, we rejected the outliers from our dataset. Outliers are abnormal values or we can say that they are deviated values from normal values. Outliers can be calculated from the following equation:

(8) $$\begin{array}{c} p\left(x\right)=\left\{x,\;\text{if }q_{1}-1.5*\text{IQR}\leq x\leq q_{3}+1.5*\text{IQR},\;\text{reject otherwise}\right., \end{array}$$

where *P* (*x*) is the mathematical formulation of outlier rejection, [11] *x* represents the instances of the feature vector that lies in the *n*-dimensional space, and *q*_1_, *q*_3_, and IQR are the first quartile, third quartile, and interquartile ranges of the attributes. After rejection of outliers, data were subjected to filling missing values. There are too many null observations in the dataset which can lead to false prediction of the patient. We have imputed the missing values by mean filter. Imputation of missing values by mean does not introduce outliers either.

(9) $$\begin{array}{c} q\left(x\right)=\left\{\text{mean}\left(x\right)\right.,\;\text{if }x=\frac{\text{null}}{\text{missed}},\;x\text{ otherwise,} \end{array}$$

where *q* (*x*) in equation (9) is the mathematical formulation of mean imputation and *x* represents the instances of the feature vector that lies in the *n*-dimensional space, where mean is calculated by averaging all the values of particular attribute. After preprocessing techniques, we have subjected our data to 10-fold cross-validation protocol in which every fold will get the chance to become trained set as well as test set. *K* − 1 set will be used as training dataset and rest 1 will be used as testing dataset. The next step is the optimization of parameters in the K-nearest neighbour, random forest, decision trees, and neural network. Parameters which are optimized for various classifiers are shown in Table 1.

### 3.4. Machine Learning System

The proposed machine learning system is shown in Figure 1. We made use of multilayer perceptron, random forest, K-nearest neighbour, and decision trees, as well as cross-validation protocol shown in Figure 2 to classify the diabetes dataset. In the feature selection method, attributes are reduced to reduce the dimensionality and to avoid the redundant features as there are many redundant features available in the dataset. After comparing three feature selection methods, we made use of correlation method to calculate the correlation amongst the features and irrelevant features are eliminated from the dataset.

## 4. Results and Discussion

### 4.1. Patient Demographics

We made use of PIMA Indians diabetes dataset whose distribution is shown in Figures 3(a)–3(f) downloaded from Kaggle and is available publicly on UCI repository. It contains data of 768 pregnant female patients, amongst which 268 were diabetic and 500 were nondiabetic. There were 9 variables present inside the dataset; eight variables contain information about patients, and the 9th variable is the class predicting the patients as diabetic and nondiabetic. The dataset consisted of outliers and missing values. In our proposed method, we have detected the outliers and removed them from the dataset. Missing values which were present inside the dataset were imputed using mean filter approach, thus leaving the dataset in a consistent state. All the experiments were done using Weka 3.9.4. The description of the dataset is shown in Table 2.

### 4.2. Results after Proposed Method

We used correlation attribute, information gain, and principal component analysis method to identify relevant features from the dataset. The results of feature selection are shown in Table 3 with 4 features and 6 features. Once the feature selection and number of features are identified, we can continue with identified feature selection method, that is, corelation attribute selection, and the number of features selected for classification is six. The results after feature selection methodologies are shown in Table 3. After feature selection, outliers were removed, missing values were imputed, and parameters were optimized. Optimization of parameters is shown in Table 1.

### 4.3. Comparison of Different Machine Learning Algorithms Using Classification Accuracy

After applying the proposed method, we have investigated that decision trees yield an accuracy of 76.07, random forest yielded **79.8**, multilayer perceptron yielded 77.60, and K-nearest neighbour yielded 78.58. The performance parameters analyzed are sensitivity, accuracy, specificity, and area under the curve. After the application of the proposed method, we can see the remarkable increase in the accuracy and the comparison is shown in Figures 4 and 5 and Table 4 as well.

### 4.4. Comparison with Benchmarking Classifier

Various techniques have been proposed in the past related to the classification of diabetes and the comparative analysis is shown in Table 5. Li et al. [39] proposed an ensemble of support vector machines, artificial neural networks, and Naïve Bayes method with taking all the features. The authors did not apply any preprocessing techniques and the ensemble of classifiers was done on raw data, thus achieving an accuracy of 58.3%. Self-organizing maps were used by Deng and Kasabov [40] and the dataset was subjected to 10-fold cross-validation protocol and achieved the classification accuracy of 78.4%. Sisodia et al. applied decision trees, support vector machines, and Naïve Bayes classifiers to predict the diabetes and in their method Naïve Bayes outshone the other methods and the classification accuracy achieved was 76.3%. Smith et al. [41] divided the dataset into training and testing datasets, where 75% of the data were taken for training and the remaining 25% were taken for testing, and they applied ADAP neural network algorithm to achieve the accuracy of 76%. Hasan et al. took six and four features into consideration and, after application of feature selection and data preprocessing technique, an ensemble of AdaBoost and extreme Gradient boost was applied on PIMA Indians diabetes dataset to classify the data into diabetic and nondiabetic and the accuracy achieved was 78.9%. Quinlan et al. [42] applied C4.5 decision tree algorithm for classification of diabetic patients and hence achieved accuracy of 71.10%. Bozkurt et al. [43] applied artificial neural network to achieve the classification accuracy of 76%. Parashar et al. [44] achieved the classification accuracy of 77.60% by application of linear discriminant analysis and support vector machines. Sahan et al. [45] achieved the accuracy of 75.87% by applying artificial immune system. Chatreti et al. proposed the implementation of discriminant analysis and achieved the accuracy of 72%. Chatrati et al. [47] removed the missing values, therefore reducing the dataset to 460 values from which 200 observations were taken as training dataset and 260 were taken as testing dataset, thus achieving the accuracy of 78%.

### 4.5. Evaluation Parameters Metrics

The following are the evaluation parameters on which predictions are made:

 
** **Sensitivity: is a term which is used to correctly identify the disease and, in our case, it is used to identify the people who are diagnosed with diabetes, that is, the number of people who tested positive
   Specificity: is a term which is used to identify healthy people, that is, those who are not suffering from diabetes or those who tested negative
   Accuracy: how accurately our method has predicted diabetic patients as diabetic and nondiabetic patients as nondiabetic
   True positive: diabetic people identified as diabetic
   False positive: nondiabetic people incorrectly identified as diabetic
   True negative: nondiabetic people correctly identified as nondiabetic
   False negative: diabetic people incorrectly identified as nondiabetic

The evaluation parameters for the classifiers are shown in Table 6 which clearly shows that random forest classifier gives the highest sensitivity, specificity, and accuracy, while the multilayer perceptron gives the highest area under the curve. Area under the receiver operating characteristics curve (ROC) plots the graph of sensitivity versus 1 − specificity. The focus of our study covered the comprehensive analysis of three feature selection methods, that is, correlation attribute evaluation, information gain, and principal component analysis, further comparing four classifiers, that is, K-nearest neighbour, decision trees, random forest, and multilayer perceptron, thus improving accuracy by preprocessing and optimizing few hyperparameters. Finally, the performances of the classifiers were evaluated using evaluation metrics such as sensitivity, specificity, and accuracy and we have shown that random forest gives highest sensitivity, specificity, and accuracy. We have got encouraging results when compared against K-nearest neighbour, decision trees, and multilayer perceptron. The limitation of this model is that specificity achieved is not satisfactory.

## 5. Conclusion

Diabetes is a silent killer and a continuing disease and it can affect different parts of the body as well. Patients are unable to produce sufficient insulin in their body because of having high glucose in the blood. Correct prediction of the diabetes can help the healthcare professionals as well as patients for proper treatment. On the basis of evaluation metrics such as sensitivity, specificity, and accuracy, we may conclude that random forest is the best classification model compared to the other classification models, that is, K-nearest neighbour, decision trees, and multilayer perceptron. Therefore, our recommendation is to use random forest with six relevant features selected from correlation attribute evaluation for the classification of diabetes data.

## Figures and Tables

**Figure 1:** Machine learning system.

**Figure 2:** Partitioning of dataset using 5-fold cross-validation [38].

**Figure 3:** ((a)–(f)) Two-dimensional distribution of PIMA Indians diabetes dataset. (a) Line plot between glucose and blood pressure. (b) Line plot between mass and pedigree function. (c) Line plot between glucose and mass. (d) Line plot between pressure and pedigree. (e) Line plot between pressure and mass. (f) Line plot between glucose and pedigree.

**Figure 4:** Line diagram of accuracy comparison.

**Figure 5:** Bar diagram of accuracy comparison.

**Table 1:** Hyperparameter optimization.

K-nearest neighbour	Random forest	Decision trees	Multilayer perceptron
Number of neighbours = 45	Size of each bag = 53	Confidence factor = 0.11	Learning rate = 0.003
Batch size = 100	Max depth = 0	Min num. of objects = 1	Momentum = 0.9
Algorithm = linear search	No. of trees = 100	Unpruned = false	Hidden layers = 10
Distance function = Manhattan function			

**Table 2:** Description of PIMA Indian diabetes dataset.

S. No	Attributes	Mean	Standard deviation	Min/max value
1	No. of times pregnant	3.8	3.4	1/17
2	Plasma glucose concentration	120.9	32	56/197
3	Diastolic blood Pressure	69.1	19.4	24/110
4	Triceps skin fold thickness (mm)	20.5	16	7/52
5	2-Hour serum insulin	79.8	115.2	15/846
6	Body mass index (kg/m^2^)	32	7.9	18.2/57.3
7	Diabetes pedigree function	0.5	0.3	0.0850/2.32
8	Age	33.2	11.8	21/81
9	Class		Tested positive:	Diabetic
			Tested negative:	Nondiabetic

**Table 3:** Accuracy of classifiers for different feature selection technique.

*N*	Algorithm	Correlation attribute	Information	Gain	Principal component
6	Multilayer perceptron	**75.1**	74.8		74.0
	Decision trees	74.3	74.2		73.5
	Random forest	**74.2**	74.6		75.1
	K-nearest neighbour	67.0	68.0		65.7

4	Multilayer perceptron	75.1	76.9		72.6
	Decision trees	74.0	74.3		72.5
	Random forest	73.3	71.7		72.3
	K-nearest neighbour	70.1	68.0		65.7

**Table 4:** Comparison of accuracy after proposed system.

S. no.	Classification algorithm	Before	Proposed method	After proposed method
1	K-nearest neighbour		70.1	78.58
2	Random forest		75.9	**79.83**
3	Decision trees		73.8	76.07
4	Multilayer perceptron		75.1	77.60

Bold means the improved accuracy after the proposed method.

**Table 5:** Classification accuracy of different methods with literature.

Authors	Data size	Techniques	Classification accuracy (%)
Li et al. [39]	768	Ensemble of SVM, ANN, and NB	58.3
Deng and Kasabov [40]	768	Self-organizing maps	78.40
Brahim-Belhouari and Bermak [16]	768	NB, SVM, DT	76.30
Smith et al. [41]	768	Neural ADAP algorithm	76
Choubey et al. [2]	768	Ensemble of RF and XB	78.9
Quinlan et al. [42]	768	C4.5 Decision trees	71.10
Bozkurt et al. [43]	768	Artificial neural network	76.0
Parashar et al. [44]	768	SVM, LDA	77.60
Sahan et al. [45]	768	Artificial immune System	75.87
Chatreti et al. [46]	768	Linear discriminant analysis	72
Christobel and Sivaprakasam [47]	460	K-nearest neighbour	78.16
Smith et al. [41]	768	Ensemble of MLP and NB	64.1
Proposed method	768	KNN, **RF**, DT, MLP	**79.8**

**Table 6:** Evaluation parameters.

S. no.	Classification algorithm	Sensitivity	Specificity	AUC	Accuracy
1	K-nearest neighbour	0.786	0.659	0.838	78.58
2	Random forest	**0.798**	**0.714**	0.836	**79.83**
3	Decision trees	0.761	0.691	0.785	76.07
4	Multilayer perceptron	0.776	0.679	**0.846**	77.60

Bold means the improvement in sensitivity, specificity, AUC, and accuracy after the proposed method.

## Data Availability

The dataset is publicly available on UCI Repository.

## Abbreviations:

SVM: Support vector machines
ANN: Artificial neural network
NB: Naïve Bayes
DT: Decision trees
NN: Neural network
RF: Random forest
XB: Extreme Gradient boost
LDA: Linear discriminant analysis
MLP: Multilayer perceptron
KNN: K-nearest neighbour.
